# Natural Compounds or Their Derivatives against Breast Cancer: A Computational Study

**DOI:** 10.1155/2022/5886269

**Published:** 2022-07-05

**Authors:** Rajib Hossain, Pranta Ray, Chandan Sarkar, Md. Shahazul Islam, Rasel Ahmed Khan, Abul Bashar Ripon Khalipha, Muhammad Torequl Islam, William C. Cho, Miquel Martorell, Javad Sharifi-Rad, Monica Butnariu, Almagul Umbetova, Daniela Calina

**Affiliations:** ^1^Department of Pharmacy, Life Science Faculty, Bangabandhu Sheikh Mujibur Rahman Science and Technology University, Gopalganj 8100, Bangladesh; ^2^Department of Biomedical Engineering, Huazhong University of Science and Technology, Wuhan, China; ^3^Pharmacy Discipline, Life Science School, Khulna University, Khulna 9280, Bangladesh; ^4^Department of Clinical Oncology, Queen Elizabeth Hospital, 30 Gascoigne Road, Hong Kong 999077, China; ^5^Department of Nutrition and Dietetics, Faculty of Pharmacy, and Centre for Healthy Living, University of Concepción, 4070386 Concepción, Chile; ^6^Facultad de Medicina, Universidad del Azuay, Cuenca, Ecuador; ^7^Banat's University of Agricultural Sciences and Veterinary Medicine “King Michael I of Romania” from Timisoara, Romania; ^8^Faculty of Chemistry and Chemical Technology, Al-Farabi Kazakh National University, 050040 Almaty, Kazakhstan; ^9^Department of Clinical Pharmacy, University of Medicine and Pharmacy of Craiova, 200349 Craiova, Romania

## Abstract

**Background:**

Breast cancer is one of the most common types of cancer diagnosed and the second leading cause of death among women. Breast cancer susceptibility proteins of type 1 and 2 are human tumor suppressor genes. Genetic variations/mutations in these two genes lead to overexpression of human breast tumor suppressor genes (e.g., BRCA1, BRCA2), which triggers uncontrolled duplication of cells in humans. In addition, multidrug resistance protein 1 (MDR1), an important cell membrane protein that pumps many foreign substances from cells, is also responsible for developing resistance to cancer chemotherapy. *Aim of the Study*. The aim of this study was to analyze some natural compounds or their derivatives as part of the development of strong inhibitors for breast cancer. *Methodology*. Molecular docking studies were performed using compounds known in the literature to be effective against BRCA1 and BRCA2 and MDR1, with positive control being 5-fluorouracil, an antineoplastic drug as a positive control.

**Results:**

The binding affinity of the compounds was analyzed, and it was observed that they had a better binding affinity for the target proteins than the standard drug 5-fluorouracil. Among the compounds analyzed, *α*-hederin, andrographolide, apigenin, asiatic acid, auricular acid, sinularin, curcumin, citrinin, hispolon, nerol, phytol, retinol palmitate, and sclareol showed the best binding affinity energy to the BRCA1, BRCA2, and MDR1 proteins, respectively.

**Conclusions:**

*α*-Hederin, andrographolide, apigenin, asiatic acid, auricular acid, hispolon, sclareol, curcumin, citrinin, and sinularin or their derivatives can be a good source of anticancer agents in breast cancer.

## 1. Introduction

Breast cancer is one of the common types of diagnosed cancers and the second prime cause of death among women in western countries [1] and develops from breast tissue [2]. Most of the breast cancers are sporadic (90-95%); between 5 and 10% can be attributed to genetic predisposition with patients having a strong family history of the disease [3, 4]. These hereditary breast cancers, a large part about 80-90% cases, are related to germ line mutations within the *BRCA1*, *BRCA2*, and *MDR1* gene [5–9]. By DNA repairing, cell cycle control and transcriptional regulation *BRCA1* may contribute to its tumor suppressor activity [10, 11].

BRCA1 and BRCA2 are also human tumor suppressor genes [6, 12], designed to chromosome 17q21 which encodes a nuclear protein of 1863 amino acids [9] that regulate transcriptional activation, DNA repair, apoptosis, cell-cycle checkpoint control, and chromosomal remodeling [13]. On the other hand, *BRCA2* located to chromosome 13q12-q13 [14] and coding for a protein of 3418 amino acids [15, 16]. Of the breast cancer susceptibility genes which have been identified nowadays, BRCA1 and BRCA2 are the most fundamental “high-risk” genes with several cases of breast and ovarian cancer accounting for most of the families [17]. If *BRCA1* or *BRCA2* is damaged by a BRCA mutation, damaged DNA is not repaired properly, and this increases the risk for breast cancer [18, 19]. P-glycoprotein 1 (P-gp1), encoded by multidrug resistance protein 1 (MDR1), is an important protein of the cell membrane that pumps many foreign substances out of cells.

Most of the initially responsive breast tumors acquire a multidrug resistance phenotype [20, 21]. The development of a multidrug-resistant phenotype in metastatic breast cancer is primarily responsible for the failure of current treatment regimens [22, 23]. Resistance to multiple drugs (MDR) is defined as efflux activity, which may decrease intracellular chemotherapeutic concentrations, thus explaining the failure of treatment in human cancers [24, 25]. Consequently, P-gp overexpression is one of the main mechanisms behind decreased intracellular drug accumulation and development of MDR cancers [25, 26].

One efficient approach used to screen potential active compounds against specific target proteins, such as BRCA1 [27], BRCA2 [28] and MDR1 [29], is molecular docking simulation [30–37]. Therefore, these are important target for the design of potential anticancer activity.

## 2. Computational Methods

### 2.1. In Silico Prediction of Activity Spectra for Substances (PASS)

Prediction of anticancer activity of 16 natural compounds was done with the help of computer program, PASS (prediction of activity spectra for substances). Software estimates predicted activity spectrum of a compound as probable activity (Pa) and probable inactivity (Pi) [38]. The prediction of activity is based on structure-activity relationship analysis of the training set containing more than 200,000 compounds exhibiting more than 3800 kinds of biological activities. The values of Pa and Pi vary between 0.000 and 1.000. Only activities with Pa > Pi are considered as possible for a particular compound. If Pa > 0.7, the probability of experimental pharmacological action is high and if 0.5 < Pa < 0.7, probability of experimental pharmacological action is less. If the value of Pa < 0.5, the chance of finding the activity experimentally is less, but it may indicate a chance of finding a new compound [39–41].

### 2.2. Ligand Preparation

The main phytochemicals and one approved drug for breast cancer treatment were downloaded from PubChem in the SDF file format. PubChem is a database for chemical molecules [42] (Figure 1).

The system is maintained by the National Centre for Biotechnology Information (NCBI), a component of the National Library of Medicine. By using Gaussian view 09 and Chem3D Pro12.0 program packages [43], all internal energies of the ligands were optimized.

### 2.3. Protein Collection

The crystal structures of proteins including BRCA1 (4Y2G) [27], BRCA2 (3EU7) [28], and MDR1 (6C0V) [29] (Figure 2) were collected from the Protein Data Bank (PDB) database [44]. For the purpose of energy minimization crystal structure, we utilized Swiss-PDB Viewer software package (version 4.1.0), and then, all the heteroatoms and water molecules of proteins are removed by using PyMOL (version 1.7.4.5) before docking [45]. Both the proteins and drug structures, for the analysis of docking results, are taken into PDBQT format finally [46].

### 2.4. Docking Analysis and Determination of Binding Site

In *in silico* study, molecular docking is a brilliant instrument which is used for predicting the drugs candidate's pharmacodynamics profile by scoring and orienting them to the receptor binding sites [47]. Docking result determines the measure of ligand interaction to the active site of the targeted protein. The docking outcome specifies the degree of ligand interaction with the desired protein's active site. The active binding sites of the target protein are the locations of the ligand in the initial target protein grids (40 × 40 × 40), with PyMOL, AutoDock Vina [48, 49], and the active sites are the coordinates of the target protein ligand, and these active target protein binding sites were analyzed using Drug Discovery Studio version v.20.1.0.19295 and 3D Ligand Site Virtual Tool [50, 51].

## 3. Results and Discussion

### 3.1. Binding Energy of the Ligand-Protein Complex

The docking is essential to predict the stronger binder and virtually screen a database of compounds. The compounds *α*-hederin, andrographolide, apigenin, ascorbic acid, asiatic acid, auricularic acid, citrinin, curcumin, hispolon, nerol, phytol, retinol palmitate, sclareol, sinularin, thymol, thymoquinone, and 5-fluorouracil displayed binding energy including -6.9, -6.2, -6.2, -5.1, -6.5, -6.8, -7.5, -7.2, -7.8, -4.8, -4.9, -5.8, -9.8, -6.5, -5.2, -5.2, and -4.6 (kcal/mol), respectively, against BRCA1 (4Y2G). Here, asiatic acid had the highest binding energy compared to the other compounds.

On the contrary, *α*-hederin, andrographolide, apigenin, ascorbic acid, asiatic acid, auricularic acid, citrinin, curcumin, hispolon, nerol, phytol, retinol palmitate, sclareol, sinularin, thymol, thymoquinone, and 5-fluorouracil, against BRCA2 (3EU7), exhibited binding energy including -11.0, -8.2, -7.7, -5.8, -8.9, -7.8, -7.6, -6.7, -6.7, -5.8, -6.4, -6.1, -7.2, -9.0, -6.5, -6.4, and -5.0 (kcal/mol). In this case, *α*-hederin produced the highest binding energy compared to the other compounds.

Moreover, *α*-hederin, andrographolide, apigenin, ascorbic acid, asiatic acid, auricularic acid, citrinin, curcumin, hispolon, nerol, phytol, retinol palmitate, sclareol, sinularin, thymol, thymoquinone, and 5-fluorouracil showed binding energy including -8.3, -9.2, -9.0, -6.3, -8.1, -8.5, -7.6, -8.3, -7.4, -5.6, -6.0, -6.2, -6.8, -8.4, -6.7, -7.4, and -5.2, respectively, against MDR1 (6C0V) (Table 1). The compound andrographolide displayed the highest binding energy compared to the other compounds.

### 3.2. Interaction and Binding Affinity of Compounds towards BRCA1 (4Y2G) Protein

Here, the ten best natural compounds such as sclareol, hispolon, citrinin, curcumin, *α*-hederin, andrographolide, apigenin, auricularic acid, and sinularin exhibited the binding affinities -9.8, -7.8, -7.5, -7.2, -6.9, -6.2, -5.8, -6.2, -6.8, and -6.5 kcal/mol (Table 2), respectively. Sclareol generated higher binding energy compared to the other derivatives against BRCA1 (4Y2G). The noncovalent interactions were calculated using Discovery Studio Software demonstrated that all the compounds exhibited both hydrogen and hydrophobic bonds that not only promoted the binding affinity but also improved binding specificity.

The compound, sclareol, showed strong hydrogen bonding with Lys1702 and hydrophobic interactions with Leu1657, Leu1679, Pre1662, Pro1659, and Val1654 residues but hispolon and citrinin exhibited only one strong H-bond with Arg1758, Arg1762, Val1654, and leu1657, respectively, as well as hydrophobic interactions with Ile1760 and Ser1755 for hispolon and with Phe1662 for citrinin. Curcumin exhibited one hydrogen bond with leu1657 and one hydrophobic bond with Phe1662, whereas 5FU exerted four H-bonds (Gly1656, Leu1657, Lys1702, and Val1654) and other hydrophobic interactions (Phe1662) with BRCA1. The other compounds have several hydrophobic interactions with BRCA1 protein residues (Table 2). The 2D and 3D structures of nonbond interactions are given in Figure 3.

### 3.3. Interaction and Binding Affinity of Compounds towards BRCA2 (3EU7) Protein

The binding affinities of *α*-hederin, andrographolide, asiatic acid, sinularin, auricularic acid, apigenin, citrinin, sclareol, curcumin, and hispolon are -11.0, -8.2, -8.9, -9.0, -7.8, -7.7, -7.6, -7.2, -6.7, and -6.7 kcal/mol (Table 3), respectively. In comparison to *α*-hederin, the other compounds showed lower binding results and *α*-hederin exhibited -11.0 kcal/mol against BRCA2 (3EU7). The nonbond interactions using the Discovery Studio Software suggested that these compounds with BRCA2 have both hydrogen and hydrophobic interactions (Figure 4) that successfully augmented the binding interactions. We found six strong hydrogen bonds (Table 3) including carbon and conventional H-bonds with amino residues including Val925, Val928, His1061, Pro926, Gly1166, and Ala874 in the *α*-hederin compound; four hydrogen bonds with Gln1020, Gly1021, Leu1143, and Leu1142 in andrographolide; and two hydrogen bonds with GLY1166 and VAL1123 in asiatic acid. In *α*-hederin, several hydrophobic interactions such as alkyl bonds were observed with Leu970, Lys1062, and Pro924.

On the other hand, andrographolide exhibited one pi-sigma bond with Phe1071 as well as alkyl and pi-alkyl with Leu1092 and Tyr1064 residues. Besides, asiatic acid generated two alkyl bonds with Pro924 and Pro926. Sinularin had several hydrophobic interactions with Leu1143, Val1073, Leu1092, Leu1142, Tyr1064, and Phe1071 residues (Figure 4). The 2D and 3D structures of nonbond interactions are given in Figure 4.

### 3.4. Interaction and Binding Affinity of Compounds towards MDR1 (6C0V) Protein

The binding affinities of these six compounds including *α*-hederin, andrographolide, apigenin, asiatic acid, auricularic acid, and sinularin, curcumin, citrinin, hispolon, thymoquinone are -8.3, -9.2, -9.0, -8.5, -8.1, -8.4, -8.3, -7.6, -7.4, and -7.4 kcal/mol, respectively (Table 4). Among those compounds, the andrographolide exhibited significantly improved binding energy compared to the other compounds binding with MDR1 protein. Herein, the nonbond interactions were performed by utilizing the Discovery Studio Software and we found that both drugs had efficient interactions with amino acid residues and both drugs showed strong hydrogen bonding (Table 4) with amino residues (Figure 5) including *α*-hederin with Lys48 and Met51; andrographolide with Ser434, Gln475, and Leu1176; apigenin with Tyr310; and auricularic acid with Lys234.

These hydrogen bonds promoted the nonbond interactions. Beyond the H-bond interactions, hydrophobic interactions play a crucial function in nonbond interaction and in this study, we observed several hydrophobic interactions (Table 4) and the residues including ALA233, ILE352, ILE190, PHE37, TRP136, PHE193, PHE194, and PHE355 with *α*- hederin; Thr906, Asn903, and Arg905 with andrographolide; PHE728, PHE732, LEU339, PHE335, PHE759, and LEU339 with apigenin; Ala233, Ile352, Ile190, Phe37, Phe193, Phe194; and Phe355 with auricularic acid. The 2D and 3D structures of nonbond interactions are given in Figure 5.

## 4. Conclusion

It can be concluded from the overall study that *α*-hederin, andrographolide, apigenin, asiatic acid, auricularic acid, and sinularin have potent inhibitory activity against cancer proteins (BRCA1, BRCA2, and MDR1) compared to the other compounds. All the compounds exhibited significant binding energies and the noncovalent bonds compared to the other compounds. Nevertheless, *α*-hederin, andrographolide, apigenin, asiatic acid, auricularic acid, and sinularin successfully docked with BRCA1, BRCA2, and MDR1 proteins as these compounds have the activity for inhibiting cancer. The nonbonding interactions can effectively target the proteins for the inhibition of cancer. We have claimed from the overall studies that *α*-hederin, andrographolide, apigenin, asiatic acid, auricularic acid, and sinularin will be the best conformer for BRCA1, BRCA2, and MDR1-conduced cancer for the future researchers. Our findings, in this way, could be manifested in clinical practice.

## Figures and Tables

**Figure 1:** The chemical structure of the screened compounds.

**Figure 2:** The three-dimensional structure of (a) BRCA1 (4Y2G), (b) BRCA2 (3EU7), and (c) MDR1 (6C0V).

**Figure 3:** The four best docking results for the best screened compounds with BRCA1 (PDB: 4Y2G) protein.

**Figure 4:** Docking results for the four best screened compounds with BRCA2 (3EU7) protein.

**Figure 5:** The four best docking results for screened compounds with MDR1 (6C0V) protein.

**Table 1:** Docking results for some natural compounds against BRCA1, BRCA2, and MDR1 proteins.

Compounds	BRCA1 (4Y2G)	BRCA2 (3EU7)	MDR1 (6C0V)
*α*-Hederin	-6.9	-11.0	-8.3
Andrographolide	-6.2	-8.2	-9.2
Apigenin	-6.2	-7.7	-9.0
Ascorbic acid	-5.1	-5.8	-6.3
Asiatic acid	-6.5	-8.9	-8.1
Auricularic acid	-6.8	-7.8	-8.5
Citrinin	-7.5	-7.6	-7.6
Curcumin	-7.2	-6.7	-8.3
Hispolon	-7.8	-6.7	-7.4
Nerol	-4.8	-5.8	-5.6
Phytol	-4.9	-6.4	-6.0
Retinol palmitate	-5.8	-6.1	-6.2
Sclareol	-9.8	-7.2	-6.8
Sinularin	-6.5	-9.0	-8.4
Thymol	-5.2	-6.5	-6.7
Thymoquinone	-5.2	-6.4	-7.4
5-Fluorouracil	-4.6	-5.0	-5.2

**Table 2:** Docking results for the best binding affinity with BRCA1 (4Y2G) protein for ten compounds.

Drug	Binding affinity (kcal/mol)	No. of H-bond	Residues
Sclareol	-9.8	1	Lys1702, Leu1657, Leu1679, Pre1662, Pro1659, Val1654
Hispolon	-7.8	2	Arg1758, Arg1762, Ile1760, Ser1755
Citrinin	-7.5	2	Val1654, leu1657, Phe1662
Curcumin	-7.2	1	leu1657, Phe1662
*α*-Hederin	-6.9	2	VAL1810, GLU1836, PRO1812, ILE1855, PHE1821, HIS1822
Andrographolide	-6.2	2	PRO1659, LEU1657, PHE1662
Apigenin	-5.8	1	LEU1657, PHE1662, VAL1654, PRO1659
Auricularic acid	-6.2	0	PHE1662, VAL1654, PRO1659
Sinularin	-6.8	1	LEU1657, PHE1662
Asiatic acid	-6.5	2	Leu1657, Lys1702, Phe1662
5-Fluorouracil	-4.5	4	Gly1656, Leu1657, Lys1702, Val1654, Phe1662

**Table 3:** The ten best docking results for the best binding affinity with BRCA2 (3EU7) protein.

Drug	Binding affinity (kcal/mol)	H-bond	Residues
*α*-Hederin	-11.0	6	Val925, Val928, His1061, Pro926, Gly1166, Ala874, Leu970, Lys1062, Pro924
Andrographolide	-8.2	4	Gln1020, Gly1021, Leu1143, Leu1142, Phe1071, Leu1092, Tyr1064
Asiatic acid	-8.9	2	Gly1166, Val1123, Pro924, Pro926
Sinularin	-9.0	0	Leu1143, Val1073, Leu1092, Leu1142, Tyr1064, Phe1071
Auricularic acid	-7.8	0	Leu1092, Leu1143, His1126, Phe1071, Tyr1064
Apigenin	-7.7	3	Asp927, Val928, Trp1164,Lys1124, Pro824, Pro926
Citrinin	-7.6	2	Gln1020, Glu1066, Leu1092, Leu1142, leu1143, Phe1071, Tyr1064
Sclareol	-7.2	1	Leu1142, Leu1092, leu1143, Phe1071, Tyr1064
Curcumin	-6.7	1	Glu1066, leu1143, Phe1071, Tyr1064
Hispolon	-6.7	3	Gly1166, Val925, Val928, Met875
5-Fluorouracil	-5.0	3	Val925, Val928, Asp927

**Table 4:** The ten best docking results for the best binding affinity with MDR1 (6C0V) protein.

Drug	Binding affinity (kcal/mol)	H-bond	Residues
*α*-Hederin	-8.3	2	LYS48, MET51, ALA233, ILE352, ILE190, PHE37, TRP136, PHE193, PHE194, PHE355
Andrographolide	-9.2	4	SER434, THR906, GLN475, LEU1176, ASN903, ARG905
Apigenin	-9.0	1	TYR310, PHE728, PHE732, LEU339, PHE335, PHE759, LEU339
Auricularic acid	-8.5	1	LYS234, ALA233, ILE352, ILE190, PHE37, PHE193, PHE194, PHE355
Asiatic acid	-8.1	3	GLU564, SER1071, VAL1052, PHE512
Sinularin	-8.4	3	GLN1118, GLU1119, SER1117, ALA529, LYS536
Curcumin	-8.3	3	Arg905, Asp1171, Lys1172, Val168
Citrinin	-7.6	2	Asp164, Arg905, Asp1124, Val168
Hispolon	-7.4	2	His166, Phe904, Phe163, Thr1174
Thymoquinone	-7.4	1	Phe904, PHE194, PHE355, Asp1124, Val168
5-Fluorouracil	-5.2	4	Arg905, Glu902, Ile901, Phe904, Phe163, Val168

## Data Availability

The data used to support the findings of this study are available from the corresponding author upon request.

## Abbreviations

BRCA1: Breast tumor suppressor gene 1
BRCA2: Breast tumor suppressor gene 2
MDR: Multiple drug resistance
MDR1: Multidrug resistance protein 1
PASS: Prediction of activity spectra for substances
P-gp: P-glycoprotein.
